# Realization of Music-Assisted Interactive Teaching System Based on Virtual Reality Technology

This article has been retracted.

**DOI:** 10.1155/2022/1007954

**Published:** 2022-06-11

**Authors:** Yan Gao, Lin Gao

**Affiliations:** ^1^Shanxi University, Taiyuan Shanxi, 030006, China; ^2^University of South Seoul, Cheonan 3102091, Republic of Korea

## Abstract

Virtual reality technology has attracted researchers' attention because it can provide users with a virtual interactive learning environment. Based on the theory of virtual reality technology, this paper proposes the system model design and architecture of virtual interactive music-assisted interactive teaching and realizes key technologies such as modeling, music-assisted interactive teaching scene interaction, and database access. In the simulation process, based on the VRML/X3D bottom interactive system template, after comprehensive application research, comparative analysis of various modeling methods, the system verified the use of digital cameras combined with the modeling technology based on music elements to collaboratively establish VRML virtual model connections. For inline node function, we combined it with Outline3D to realize VRML integration and then use VizX3D, X3D-Edit to build X3D model and realize the conversion from VRML to X3D, which solves the system completeness problem of music-assisted interactive teaching. The experimental results show that, according to the statistical analysis of the data after the experiment, when the position changes in the virtual 3D music-assisted interactive teaching scene, it will be displayed in the plane layer, and the real-time coordinates of the virtual music-assisted interactive teaching scene displayed in HTML have case. By analyzing the scenes and dynamic effects in the works, the effects of the virtual world can be better displayed through the performance of details. The better accuracy and delay error reached 89.7% and 3.11%, respectively, which effectively improved the effect and feasibility of applying virtual reality technology to music-assisted interactive teaching.

## 1. Introduction

Virtual reality technology is one of the hot areas of research at home and abroad and has played an active auxiliary role in the field of music-assisted interactive teaching [1–4]. Under the guidance of the constructivist music-assisted interactive teaching theory, it is connected with various technical means of multimedia technology and network technology, combined with the discipline of music-assisted interactive teaching, and helps learners to construct a learning environment in the virtual music-assisted interactive teaching scene. The environment and the construction of meaning are the new learning methods of interactive teaching in the new era. Constructivist learning theory emphasizes the central position of students, the important role of rich “situations” in meaning construction, and the important role of multiple learning music-assisted interactive teaching scenarios [5–7]. The virtual reality technology provides a technical guarantee for the realization of a simulated work and learning environment, which is deeply in line with the constructivist learning theory [8–11]. In the current situation at home and abroad, we can fully understand the wide range of virtual technology applications and lead the pace of the information age. The learners can interact with the learning situation through the simulation of the interactive teaching environment assisted by music, so as to realize the autonomous learning in the interactive teaching mode.

Radianti et al. [12] believes that the use of virtual reality technology in music-assisted interactive teaching can fully mobilize the learner's senses and thinking organs, so that the observed scenery is vividly displayed in front of them. Especially for some inaccessible music-assisted interactive teaching or experimental content, through virtual reality technology, they can be placed in front of them like real objects and can be carefully observed from the front, side, and back, and even inside the scene for observation and research. Odrekhivskyy et al. [13] believed that for the scenes that are difficult to restore in the real music-assisted interactive teaching, the reproduction of state can also be realized by means of virtual reality technology. Aithal and Aithal [14] found that in the music-assisted interactive teaching experiment, virtual reality can also be integrated with other multimedia technology to play a greater role. The so-called “interactivity” means that the human-computer interaction in the virtual reality system is a nearly natural interaction. Users can not only interact with a computer keyboard and mouse but also through special helmets, data gloves, and other sensing devices. Chen et al. [15] believe that the computer can adjust the musical elements presented by the system and the auxiliary interactive musical elements according to the movements of the user's head, hands, eyes, language, and body. Users can inspect or operate objects in the virtual environment through their natural skills such as language, body movements, or actions. The information felt by the user in the virtual world, through the thinking and analysis of the brain, forms the action or strategy that they want to implement, and feeds it back to the system through the input interface to realize the function of interacting with the system and independently controlling the operation of the system [16–21].

This paper starts with constructivist learning theory. From the learning point of view of learning, it analyzes the important role of virtual reality technology in the field of music-assisted interactive teaching, introduces what virtual reality technology is, the current application and development of virtual reality, VRML (virtual reality modeling language) to build the common technical means in the virtual reality music-assisted interactive teaching scene, and explain in detail the role and significance of the design in the author's actual work. Secondly, starting from the completed music-assisted interactive teaching media simulation system, the key technologies used to complete the system and the design ideas of the system are expounded, and the specific methods for completing the model making of the virtual system and optimizing the model through 3DS MAX are expressed. In the process of establishing a virtual music-assisted interactive teaching environment, the process of using VRMLPad to interact with the established music-assisted interactive teaching environment model is explained, and the music-assisted interactive teaching equipment model established by Cult3D on 3DS MAX is explained for ideas and methods for interaction. The system implemented in this paper can become an effective supplementary means of music-assisted interactive teaching in the course music-assisted interactive teaching and can help students achieve digital learning.

## 2. Methods

### 2.1. Virtual Reality Level

The Script node in the system hierarchy transmits the value of the VR event to the script specified by the URL. If it accepts a group of trigger events, the Script node processes it in sequence according to different methods. If using JavaScript, each input event corresponds to a custom function of the same name. The browser calls the functions according to the order [22]

(1) $$\begin{array}{c} \frac{d\psi^{\prime }\left(x\right)dx-d\psi^{\prime }\left(y\right)dy}{dx+dy}-\frac{d\psi^{\prime }\left(x\right)dx}{d\psi^{\prime }\left(y\right)dy}=0. \end{array}$$

This method can effectively help the file creator to easily complete the establishment of more complex models and music-assisted interactive teaching scenarios, without involving a large number of code problems, directly use the various controls integrated in the visual editor to complete the corresponding operations. During the establishment of this system, a large number of this method was used to complete the establishment of models and music-assisted interactive teaching scenarios [23–26].

Action and autonomy are inseparable from the user and the things in the scene. Whether it is a single dynamic or mutual dynamic, it is inseparable from the interaction generated by each other, because these two characteristics are also derived from the interaction. Character-assisted interaction is an auxiliary interaction mode in the virtual-assisted interaction system. The user is incarnated as an animated character in the virtual environment, and a third-person camera is placed behind the character as the user's viewpoint. The user can use the keyboard to control the movement of the character and then move the viewpoint. Character assistant interaction is a freer assistant interaction mode, which can break the limitation of automatic assistant interaction on the time and space perspective. In this example, a typical process of writing a 3D event using a text editor is illustrated. From defining a geometric model, to adding trigger nodes, to adding script events, the writing process of VRML is described.

### 2.2. Music-Assisted Dependency

The storage of data or code, in the design method for music auxiliary objects, data, or code is a whole, this whole is the object, the member data or member functions of the thorn elephant can be hidden as needed, and other objects cannot directly modify the column. Like all the data, but to be modified through the member function of this strip, so as to avoid the mutual interaction of program modules. It uses descriptive text language to describe the shape of basic three-dimensional objects and combines these basic three-dimensional shapes into a virtual music-assisted interactive teaching scene through certain control interpretation and execution to generate virtual three-dimensional music-assisted interactive teaching scenarios. The biggest feature of VRML is the use of text to describe the three-dimensional space, which greatly reduces the amount of data transmitted on the Internet.

When the sweeping stroke is many polygons of the environment of Figure 1, its capture transformation process polygon is similar. But at this time, there is a mutual occlusion relationship between polygons, so it is necessary to determine and calculate the visible scan line segments in each scan line, that is, to perform blanking processing. This process can be divided into two steps: calculating the scan line segment and determining the visibility of the line segment. The first step is to calculate.

(2) $$\begin{array}{c} \frac{dx\left(i,j\right)}{didj}=\frac{x\left(i\right)/x\left(j\right)}{x\left(j\right)-1}-\frac{\left(1-i-j\right)x}{x\left(i\right)-1}. \end{array}$$

All intersecting line segments of the sweep line and the polygon formed by the object in the auxiliary interactive music elements. The second step eliminates the invisible line segment or part of the line segment.

### 2.3. Music-Assisted Interactive Teaching Media

Routing is the connection channel between the nodes that generate music auxiliary events and receive events, and the routing of events ROUTE can make VRML programs interactive. The routing transmits the events generated by some nodes to other nodes, and, by changing the attribute values of some fields, makes the objects in the three-dimensional space produce motion or special effects, that is, animation and interaction, making the virtual world more realistic. The sense of presence in virtual reality itself is the thing that exists, and the sense of presence is the real feedback that the real thing can give the experiencer. The virtual scene itself is built on the basis of the real thing.

The music element program algorithm of the system loading music auxiliary interface is basically the same as that of the main interface. However, its highlight is that when the system loads the music-assisted interactive teaching scene, the operation instruction display function is added, which not only allows the user to understand the specific operation steps while waiting but also diverts the user's attention and ignores the waiting time, thus strengthening the user sensory experience. In the process of auxiliary interactive programming, in order to reduce the model burden of the system, when the music-assisted interactive teaching scene is loaded into the program design, we store the music-assisted interactive teaching scene in a Virtools file in Table 1, according to the auxiliary interaction selected by the user. Patterns are dynamically added to the system.

It is used in conjunction with the *f* frame buffer to complete the blanking function. The initial value of each unit in the *z* buffer is taken as the background color or gray value of the corresponding picture. Musical element blanking is achieved during the drawing of the musical element. When the image is drawn, when the attribute (color or grayscale) value of each pair (pixel) of the display wipe is filled into the corresponding unit of the frame buffer, the *z*-coordinate value of the point should be corresponding to the *z*-buffer. The values within the cell are compared. If the former is greater than the latter, change the value of the corresponding unit of the frame buffer and update the value of the corresponding unit of the *z*-buffer to this, and draw the *z*-coordinate of the gate. On the contrary, if the *z*-coordinate value of the point is smaller than that of the corresponding unit in the *z*-buffer value, it means that the point is farther from the viewer than the displayed point and is therefore occluded.

## 3. Results

### 3.1. Virtual Reality Data Pooling

In the process of completing the construction of the virtual music-assisted interactive teaching environment, after completing the model, save the file format as wrl, and add interaction. In the modeling of each music-assisted interactive teaching equipment, it is convenient to use VRMLPAD to modify it later. Since there are a lot of interactive processes in this part, it will be a very huge project if the VRML language is written manually. Therefore, we choose to use CULT3D for interactive designs. For this part, save the established equipment model in 3DMAX as the C3D format shown in Figure 2 to facilitate the use of subsequent steps. Combined with the relevant experimental data of inverse kinematics, the key frames are simulated to achieve three-dimensional modeling and display, which can intuitively reproduce the standard technical movements of athletes and provide key elements for course teaching.

The material has four property settings: ambient, diffuse, specular, and emissive, which represent ambient light, diffuse reflection light, and specular reflection properties, respectively. Emissive represents the luminosity of the auxiliary interactive music element light itself. The four parameters are all values of type color. There is also a power property, which is a floating point type. The larger the value, the greater the difference between the highlight intensity and the surrounding brightness. The parallel line parallel to the coordinate axis, the vanishing point formed on the surface of the auxiliary interactive musical element is called the main vanishing point. According to the number of main vanishing points, perspective auxiliary interactive music elements are further divided into one-point perspective, two-point perspective, and three-point perspective. Compared with the parallel auxiliary interactive music elements, the perspective auxiliary interactive music elements have a stronger sense of depth and look more realistic. But perspective projection cannot truly reflect the exact size and shape of objects.

Students' movements can also be recorded through sensors and motion sensing devices, and the comparison of data differences can be used to judge the standardization of students' movements and realize the interaction between the virtual world and the real world. The higher the sample rate and resolution of the auxiliary interactive musical elements, the more memory is consumed when the auxiliary interactive musical elements file is loaded into the computer. Not all sound cards can support high sampling rates and whether it is necessary to use high sampling rate auxiliary interactive music elements, because human ears are not that powerful, too high resolution is just a waste of memory. In order to save memory and improve the efficiency of the CPU, the virtual auxiliary interactive system uses the auxiliary interactive music element stream to process the music module, that is, the auxiliary interactive music element file is streamed. The principle is this: first load the first point of the auxiliary interactive music element file into the memory, and then load the rest of the file into the memory one after another during playback.

### 3.2. Music Helper Function Recursion

In the function recursion of computer music elements, the homogeneous coordinate technique is widely used to study the transformation of music elements, that is, in the *n* + 1 dimensional space, the transformation of *n*-dimensional vectors is discussed, and the normalization process is performed to observe its transformation in the *n*-dimensional space result. It is precisely because the geometric transformation of music elements can be transformed into the multiplication of a vector representing the point set of music elements and a certain transformation matrix, so the transformed music elements can be obtained quickly, which provides the possibility for the dynamic display of computer music elements. No matter in the two-dimensional plane or the three-dimensional space, the defined geometric musical elements can be continuously transformed for many times to obtain the new required musical elements. At this time, it is only necessary to multiply the corresponding multiple transformation matrices to form a combined transformation matrix, and then act on the geometric music elements.

(3) $$\begin{array}{c} X\left(\text{a},\text{b}\right)=\left[\begin{array}{ccc} \psi^{\prime }\left(\text{a}\right)da & 1-a & 0\\ 1-a & \psi^{\prime }\left(\text{a}\right)da & 1-a\\ 0 & 1-a & \psi^{\prime }\left(\text{a}\right)da \end{array}\right]. \end{array}$$

It mainly calculates the specific direction and specific position of the tracked object by using the video camera to reach the *X*-*Y* plane array, the surrounding light or the projection of the tracking light in the projection plane at different times and different positions. Making a path curve function in Virtools is composed of some 3D nodes and curves. These elements can be made through functions. After they are made, they can be used as a path curve function after setting. The key code is introduced first. X3D's text editors mainly include X3D-Edit, an open-source X3D development tool developed by the Web3D Alliance, and X3D is also an open-source X3D development toolkit. X3D-Edit is an Extensible 3D (X3D) text editor for musical elements, edit customizes the general XML editor under the Java platform through the X3D 3.0 tagset defined by the X3D 3.0 DTD, and uses IBM Xeena as the customized X3D music-assisted interactive teaching scene graph editor. Supported platforms are Windows, MacOS X, Linux, Unix, and others. The higher the hierarchy, the system will display who is the priority. The hierarchical relationship of 2D frames can be set at any time to ensure that no logical errors will occur during the real-time display of 2D frames.

### 3.3. Deep Fit of Music-Assisted Interactive Teaching

The interactive teaching output is divided into three parts: static output, dynamic output, and online version output. Different output forms have different effects. With the support of different technologies, the effects that can be displayed are different, and there are also gaps in practical effects. There are two technical forms of virtual reality technology in works. One is operational technology, which conducts in-depth research and development through existing tools and software technology and the successful case form of previous researchers. For example, the touch-type structure, which uses the mouse and keyboard to operate the virtual space of the computer screen, is also a form of relatively traditional virtual assisted interaction technology, and it is also one of the fastest forms accepted by users.

(4) $$\begin{array}{c} \left\{\begin{array}{c} U\left(i,j\right)=u\left(i,j\right)-\frac{u\left(i\right)-u\left(j\right)}{u\left(i\right)-u\left(j\right)},\\ W\left(i,j\right)=w\left(i,j\right)-\frac{w\left(i\right)-w\left(j\right)}{w\left(i\right)-w\left(j\right)}. \end{array}\right. \end{array}$$

The main functions realized by the interactive teaching interface module design algorithm are: system initialization, loading textures, materials, and other materials; initial interface and button display; click the button to enter the corresponding function interface; function interface initialization, loading function interface materials; function interface and button display; click the button under the function interface to switch back to the initial interface; after the system is terminated, destroy the data and release the memory. When editing VRML or X3D music-assisted interactive teaching scene graph files, X3D-Edit can provide a simplified and error-free way of creating and editing, edit customizes context-sensitive tooltips through XML files, providing a summary of each node and attribute to facilitate authoring and editing of music-assisted interactive teaching scene graphs. When students use virtual reality technology, students can concentrate faster and more lastingly, the number of questions asked by teachers is relatively reduced, and the work intensity of teachers is reduced. The interactive teaching effect is unanimously optimistic. In this virtual environment, students are not students in the classroom in the biological sense, but refer to those who need to obtain learning information and resources into the virtual teaching environment, and then participate in learning activities through their avatars.

In the virtual music-assisted interactive teaching scene, except for the boundary scope of Figure 3, such as the music-assisted interactive teaching building and the music-assisted interactive teaching facilities, the characters cannot pass through. Due to the interaction between the system and the user and the movement of the character, the character and the virtual stationary object may collide. In order to maintain the authenticity of the virtual auxiliary interaction system, it is necessary to detect the possible collision in time and design the corresponding collision response; otherwise, the character will occur, which affects the realism of the auxiliary interactive system and affects the user's immersion. There are 255∗255 horizontal and vertical grids in the grid, and the value of each grid ranges from 0 to 255. When the grid value is 255, it turns yellow, indicating that the grid is forbidden to be crossed. Clever use of numerical values is to plan the limited boundary of the character's movement and calculate the straight-line distance between the character and the boundary in real time, when the distance is less than 0, stop the character's progress, indicates that the character has reached the boundary at this time. The function that bounds the character's motion is setBoundary ().

### 3.4. Parameter Configuration of Music-Assisted Interactive Teaching Scene

For the three-dimensional music-assisted interactive teaching scenes and objects displayed on the Internet, VRML is described using a file format standard, and any editor can be used as a writing tool. Analyze and discuss the role of virtual reality technology in teaching and the application of virtual reality technology in teaching, listen carefully to experts' opinions and adopt them, provide multiple perspectives to promote the research of this paper and provide more realistic basis for the paper. To enter the virtual reality world, users only need to access through the VRML browser and download the music elements music elements and audio and video resources placed on the server. In addition, VRML's rendering of musical elements is real-time as the user interacts with objects in the virtual world in real-time. VRML provides 6 + 1 degrees of freedom, that is, rotation and movement in three directions, as well as hyperlinks (Anchors) with other 3D spaces. Users can intuitively feel the impact and changes of their own behavior on the virtual world.

(5) $$\begin{array}{c} \frac{\text{Dertimerst}\left(c,c-1\right)}{c\left(x\right)}\in \left[\begin{array}{c} \left[0,1,2,\cdots ,c-1\right]\\ \left[0,1,2,\cdots ,\sqrt{c}-1\right]\\ \left[0,1,2,\cdots ,\sqrt{c-1}\right] \end{array}\right]. \end{array}$$

User domain refers to the entire natural space that programmers use to define sketches. This defines a yellow cube with length 2, width and height 1. The main attribute of the box node is size, which is used to determine the size in the length (*x* direction), height (*y* direction), and width (*z* direction). It is better to use the English folder name to save the file, because in the folder (path), you can only browse and run the files that do not use Java class and music assisted interactive teaching scene; otherwise, you cannot even see the X3D music-assisted interactive teaching scene. The windows can be nested, that is, the second layer window can be defined in the first layer window, the *i* + 1 layer window can be defined in the *i*-layer window, and so on. In some cases, the users can also define a circular window with a center and a radius or a polygonal window represented by a boundary, as needed.

## 4. Discussion

### 4.1. Extraction of Virtual Reality Factors

For VRML browsers, in theory, it can process multiple virtual reality factor objects distributed on the Internet. Enhancing the quality of the musical elements and emulations in case of poor performance, or reduce the quality of musical elements and emulations in the case of poor performance. The node “multiple levels of detail (LOD)” provided by VRML can simulate the situation observed by the human eye in reality. When the distance from an object is relatively far, the details of the object are not clear; but when the distance from the object is getting closer, the level of detail of the object is more and more clear. The selection criterion of the level of detail in VRML is the distance from the viewpoint to the geometry, and the system selects different LOD levels according to the distance. At the beginning of the formal experiment, a questionnaire survey was conducted on the application of virtual reality technology in teaching. The questionnaire was distributed through the network. After the experiment, a questionnaire survey was conducted on the students in the experimental group. When the distance is greater than or equal to a certain value of Figure 4, the observer will move to the next level of detail.

In most cases, the client and server run on the same machine, of course, it can also be used in a network environment, so OpenGL has network transparency, and the music element function library is encapsulated in the win32 music element device interface (GD) dynamic link library OpenGL. Like in DLL, the music element library of OpenGL is also encapsulated in a dynamic link library OpenGL DLL. The call of the OpenGL function released from the client application program is firstly opened by OpenGL DLL processing, and then sent to the server by winsrv. The DLL is further processed, and then passed to the win32 device driver interface (DDI), and finally, the processed music element command is sent to the video display driver.

### 4.2. Simulation of Music-Assisted Interactive Teaching System

The core part of the interactive teaching system is designed to complete all the main functions of the system, including the premusic-assisted interactive teaching scene processing method, the system interface module, the role-assisted interaction module, the automatic auxiliary interaction module, the sound effect module and the release after the system is completed. After the development of this virtual assistant interaction system is completed, it is only a primary version, and more functions will be expanded as needed. For example, the system can be imported into a tablet computer and adopted the touch screen operation mode; a database module is added to record the key of each assistant interaction, add multirole simultaneous auxiliary interactive interaction function. The powerful secondary development function of Virtools can fully meet the needs of this system expansion function. Using the index scoring method and the chart evaluation method, with a full score of 100 points, the behavior of the testee is divided into several indicators, and each indicator is assigned a certain score, total score.

The system abstracts each geometric body into a music element class according to the idea of object-oriented programming, and each interactive teaching class encapsulates the unique attributes and behaviors of the corresponding body. The music element class mainly completes the establishment of the music element model, the generation of wireframes, entity maps, material maps, and texture maps. In addition, music element transformation methods (translation, rotation, and scaling) are provided. First, the object of the simulation is a certain floor of a music-assisted interactive teaching building, which includes multiple areas such as multimedia classrooms, offices, line editing rooms, non-editing rooms, and recording keys. According to the actual size. Using AUTOCAD2004 to draw the architectural plan, and use the file-import command to import the dwg text drawing into 3DSMAX, and use the extrude modifier to build the wall after the line is drawn. The modeling process uses basic geometry for modeling.

Any area less than or equal to the screen area is called the view area. The view area can be defined by the device coordinates in the screen area. If the music elements in the window area selected by the user are to be displayed in the view area, they must also be converted into the coordinate values in the device coordinate system by the program. The view area is generally defined as a rectangle, which is defined by the coordinates of the lower left corner and the upper right corner, or by the coordinates of the lower left corner and the x and y directions of the view area: the length of the edge. The view area can be nested, and the nested level of the music element processing software is fixed. For graphics and polygon windows, users can also define circular and polygonal view areas for different applications.

### 4.3. Example Application and Analysis

For the design of interactive teaching virtual comics, the most convenient way is to generate EXE executable files, but EXE files cannot be directly generated by Virtools, and the external VirtoolsMakeExe.exe and CustomerPlayer.exe files are needed to achieve this, it may run the VirtoolsMakeExe.exe file, the following setting interface will pop up, click the designated button corresponding to the Virtools project file option, select the CMO file we have completed, and set the resolution in the window setting option. Here, we use 1366∗768, click “Generate” button; then, the generated EXE file can be run independently of the Virtools environment. The base class of music elements is used to implement operations common to all music elements, such as translation, rotation, and zoom operations of music elements, and shapeless material settings. It also contains two virtual functions: the music element drawing function Draw() and the music element storage function Save(). Then, we use mathematical methods to establish mathematical models such as charts, analyze various data and materials obtained from the investigation and scoring through mathematical statistics, and finally form quantitative conclusions.

The functions of each voxel class are roughly the same, mainly completing voxel modeling, generating various forms of 3D models, and storing the unique data of each geometric shape. For models that appear repeatedly in multiple places, if a single modeling method is used, the code of the file will be greatly increased, and the real-time performance of the virtual music-assisted interactive teaching scene will be greatly reduced. Interactive teaching techniques are used here to apply transparent textures directly to the established 2D surfaces, or onto criss-cross patches. When setting, let the 2D object automatically adjust the normal direction according to the position of the camera.

From the perspective of self-rating items, the average score was 4.68 points higher than that of the control group. Using SPSS software for *t*-test analysis, *P* = 0.002 < 0.05 and *P* < 0.01, it can be seen that there is a very significant difference. Vizx3D includes a complete 3D modeling function and the interactive editing function of music elements as shown in Figure 5. Vizx3D supports the establishment and editing of H-anim, NURBS, texture music-assisted interactive teaching scenes, and supports XML or VRML97 encoded X3D files. Through Vizx3D, users can intuitively create music-assisted interactive teaching scenes, create animations with key frames, and create music-assisted interactive teaching scene interactions through its unique system. It can output both wrl files and x3dv files.

In the tab, you can set the resolution of the virtual auxiliary interactive system. The resolution is related to the size of the design window of this system and the display effect of the published work after the system design is completed. The resolution selected by this system is 1366∗768. After adding the lights, the music-assisted interactive teaching scene is bright, but all the models seem to have no textures on them. At this time, the models are pasted with shadow maps. Go to the Meshes settings tab, double-click the mesh under Meshes to open it, and mix it, change the mode to overlay DestColor. At this time, the texture will come out, and the color will be darker. Next, we enter the corresponding material level, brighten its color, and adjust all models to the ideal state. It shows that the students in the experimental group have improved their learning and understanding of the teaching content, are more satisfied with their self-expression, improved their self-confidence and interest in dancing, and gave themselves higher scores. If the model is transparent for the texture, change the mode to mash in material. If it is a double-sided sticker, put the box behind the both sided below.

## 5. Conclusion

This paper starts from the role of virtual technology in the auxiliary interactive music teaching environment, breaks through the traditional form of expression, technology, and auxiliary interaction complement each other in the trend of digital information, and expresses the unique auxiliary interaction personality. The main research contents of this paper include the theory of virtual reality technology in the auxiliary interactive music teaching environment, the auxiliary interactive expression of virtual reality in the auxiliary interactive music teaching environment, the interactive presentation of virtual reality technology and auxiliary interaction in the auxiliary interactive music teaching environment, auxiliary interactive music, and the realization of works of virtual reality technology and auxiliary interaction in teaching environment. In order to meet the requirements for real-time rendering of music elements in real-time interaction, scientific computing visualization and dynamic simulation, reducing the number of triangle faces of the rendered entity is a key technical issue for real-time rendering of music-assisted interactive teaching scenes in the external scenic spots of the training center and the interior of the training room, the article applies the LOD technology of the real-time generation method to set the objects of the virtual music-assisted interactive teaching scene within a certain range, so that they can show different details at different viewing distances, so that the browser can take automatic switching between different levels of detail represented. The research on virtual reality technology theory and virtual reality-assisted interactive expression under the auxiliary interactive music teaching environment guides the creation of virtual design based on the theory and finds breakthroughs in the creation and summarizes new theoretical knowledge and value achievements. The development of virtual reality technology should not be hampered by equipment. More and more convenient forms can also bring the immersive experience from reality to virtuality.

## Figures and Tables

**Figure 1:** A brief description of music-assisted reliance on browsing information.

**Figure 2:** Virtual reality-assisted interactive music element data pooling.

**Figure 3:** Distribution of deep fit of music-assisted interactive teaching.

**Figure 4:** Extraction of virtual reality network environment factors.

**Figure 5:** Interactive teaching virtual display data editing.

**Table 1:** Attributes of music-assisted interactive teaching.

Music-assisted number	Experiment system data ratio			Control system data ratio		
1	0.865	0.346	0.463	0.661	0.742	0.559
2	0.396	0.719	0.127	0.318	0.338	0.295
3	0.449	0.433	0.187	0.006	0.086	0.412
4	0.770	0.764	0.824	0.807	0.525	0.673
5	0.431	0.426	0.490	0.484	0.437	0.429

## Data Availability

The data used to support the findings of this study are available from the corresponding author upon request.
